The article "Physical Therapy for at Least 6 Months Improves Motor Symptoms in Parkinson's Patients: A Meta-Analysis" was published in 2022. Journal: Comput Math Methods Med.

# Physical Therapy for at Least 6 Months Improves Motor Symptoms in Parkinson's Patients: A Meta-Analysis

**DOI:** 10.1155/2022/3393191

**Published:** 2022-07-31

**Authors:** Xiaotian Ji, Danian Lu, Qinglan Yang, Linting Xiao, Jing Wang, Gaiqing Wang

**Affiliations:** ^1^Department of Neurology, Sanya People's Hospital, West China (Sanya) Hospital, Sichuan University, Sanya 572000, China; ^2^Department of Neurology, Sanya Central Hospital (Hainan Third People's Hospital), Sanya 572000, China

## Abstract

**Objective:**

Long-term physical therapy helps to improve the motor symptoms of patients with Parkinson's disease, but the effectiveness is not clear. The purpose of this study was to evaluate the effect of long-term physical therapy on improving motor symptoms or daily activities in Parkinson's patients with drug use or discontinuation, as well as its impact on drug treatment dose. A subgroup analysis was conducted on different treatment methods to determine the most effective treatment method.

**Methods:**

The researchers independently searched databases, including PubMed, Medline, Embase, Ovid, Cochrane Library, and ISI Web of science. The search deadline was June 2022. A randomized controlled trial was conducted on Parkinson's disease patients with HY stages 1-3 who received continuous physical therapy for 6 months or more. Systematic evaluation and meta-analysis were carried out by using common clinical evaluation indicators, namely, MDS-UPDRS exercise score, daily activity (ADL) score, or LED dose. The quality of the literature was assessed using the modified Jadad scale of Cochrane's bias risk tool.

**Results:**

A total of 523 Parkinson's disease patients with HY stages of 1-3 were included in the study. The results showed that long-term physical therapy could improve patients' motor symptoms with combined antiparkinsonian drugs (*Z* = 2.61 and *P* = 0.009) and had a significant positive effect on the motor symptoms of patients with discontinued antiparkinsonian drugs (*Z* = 2.73 and *P* = 0.006). Meanwhile, it could reduce the LED dose of patients with Parkinson's disease. The difference was statistically significant (*Z* = 2.58 and *P* = 0.010).

**Conclusion:**

The results of this study indicated that physical therapy for at least 6 months or longer for patients with mild to moderate Parkinson's HY could effectively improve the motor symptoms of Parkinson's patients, whether or not combined with antiparkinson drugs. Meanwhile, long-term physical therapy reduced the LED dose of patients treated with drugs compared with patients in the control group who received short-term physical therapy, other types of intervention group, or no treatment.

## 1. Introduction

Parkinson's disease is a common and complex neurodegenerative disease. About 1.6 people in every 1000 people worldwide suffer from Parkinson's disease. The high prevalence greatly impacts patients and their families [1]. The main symptoms of Parkinson's disease (PD) are dyskinesia and motor symptoms, including bradykinesia, static tremor, rigidity, and postural and gait disorders. With the progress of the disease, these symptoms become more prominent and impact daily activities (ADL) [2, 3]. Traditionally, the treatment of Parkinson's disease is drug treatment. Still, the patient's physical function, daily activity participation, and activity ability decline with the progress of the disease, which leads to a continuous decrease in the patient's quality of life [4]. In addition, the drug effect becomes more and more limited as increasing drug dosage and progressing disease. Meanwhile, drug side effects can increase the risk of exercise complications [5]. At present, physical therapy combined with drugs has been widely used in the clinical management of Parkinson's disease [6].

Physical therapy is an intervention method that enhances muscle strength, aerobic exercise ability, balance ability, posture and gait, and body flexibility through reminders, exercise awareness strategies, and physical exercise [7]. Previous studies have shown that physical therapy has a short-term improvement effect on motor symptoms and daily activities of patients with Parkinson's disease [8–10]. However, a few evaluate the impact of long-term physical therapy on motor symptoms, daily activities, or a combined dose of drugs in patients with Parkinson's disease. Most physiotherapy widely used in the clinic is only short-term, which may be related to the lack of high-quality systematic evaluation and meta-analysis of long-term physiotherapy. Suppose long-term physical therapy is conducive to delaying motor symptoms and ADL damage, thus reducing the dosage of antiparkinson drugs. In that case, it may benefit a large number of patients. Currently, several randomized controlled trial (RCT) studies have carried out long-term physical therapy for at least 6 months or more to reveal its impact on motor symptoms, ADL, and drug dosage of PD patients [11–13]. Furthermore, previous studies on long-term physical therapy have primarily used various physical therapy measures, including compound aerobic exercise, strength exercise, multimodal exercise, or multidisciplinary treatment programs based on physical therapy [14]. However, it is not clear which type of long-term physical therapy can benefit patients the most.

In this study, data were extracted and analyzed from the long-term physical therapy randomized controlled trials that have existed for more than 6 months. This study evaluated the effect of long-term physical therapy on motor symptoms or daily activities of patients with drug use or discontinuation and its impact on drug treatment dose. We also conducted subgroup analysis on different treatment methods to determine the most effective treatment method.

## 2. Materials and Methods

### 2.1. Literature Search Strategy and Inclusion and Exclusion Criteria

Following the principle of Cochrane, 4 independent researchers conducted a comprehensive literature retrieval. Researchers independently searched the following databases: PubMed, Medline, Embase Ovid, Cochrane Library, and ISI Web of science. The search deadline was June 2022. The search keywords were “Parkinson disease” or “Parkinsonian” and “rehabilitation” or “physical therapy” or “physiotherapy” or “exercise” or “training.” The range was human-related studies. Disagreements were resolved through negotiation and discussion.

The inclusion criteria were as follows: (1) parallel randomized controlled trials; (2) the document language was English; (3) the patients included in the study were mild to moderate Parkinson's disease patients with HY (Hoehn and Yahr stage); (4) patients received physical therapy at least once a week for 6 months or more; (5) two groups of comparative intervention experiments, namely, the long-term physical therapy experimental group and the control group, where the control group could be a short-term treatment intervention group, other types of intervention group, or no treatment group; (6) data that could be extracted before and after treatment to evaluate in this study, where data included movement disorder society UPDRS (MDS-UPDRS) motor score, daily activity (ADL) score, or levodopa equivalent dose (LED); and (7) the modified Jadad scale (RCT) score ≥4.

The exclusion criteria were as follows: (1) Non-Parkinson's disease patients with tremor paralysis symptoms; (2) atypical and widely used physical therapy interventions included but were not limited to dance, Tai Chi, qigong, yoga, music, boxing, and various nerve stimulation; (3) unable to judge whether the patient is in the state of drug use; and (4) the literature types were review, case-control study, case report, and other non-randomized controlled studies.

### 2.2. Document Data Extraction

In this study, 3 researchers extracted the basic information and data of the literature that met the inclusion criteria, and a third researcher checked the data. The extracted data and characteristics included literature characteristics (author, year of publication), patient characteristics (quantity, HY disease degree classification), physical therapy, result evaluation, and drug use during the experiment were collected. According to the previously published literature review [15], the common clinical evaluation indicators, namely, MDS-UPDRS motor score, daily activity (ADL) score, or LED dose, were used. Currently, the motor and ADL scores (MDS-UPDRS) are one of the world's standard measurement standards for exercise and the daily life of PD patients [16]. The types and doses of drugs used by different patients were different. Furthermore, the levodopa equivalent dose (LED) was adopted in this paper to facilitate the statistical conversion of the dosage of patients [17].

### 2.3. Statistical Analysis

The Review Manager software (version 5.4 of the Nordic Cochrane Centre, Copenhagen, Denmark) was used for statistical analysis and forest map, thus evaluating the total effect comparison between the long-term physical therapy group and the control group. Due to the large differences between clinical and research methods between experiments, the standardized mean difference (SMD) and 95% confidence interval (CI) were calculated for continuous variables using the random effect model. The studies with clinical homogeneity were divided into subgroups to analyze the specific effects of different types of physical therapy. The Chi-square test was used for the heterogeneity test. When *P* < 0.05, the difference was considered statistically significant.

### 2.4. Document Quality Evaluation

The modified Jadad scale of Cochrane's bias risk tool was used to assess the quality, bias, and risk of eligible studies [18]. The modified Jadad scale used in the literature evaluation was a widely used scale in clinical and research [19]. The improved M-Jadad scale was divided into random sequence generation (2 points), randomized hiding (2 points), blind method (2 points), and withdrawal (1 point), with a total of 7 points. 1-3 points were recognized as low-quality research, and 4-7 points were recognized for high-quality research. In addition, Cochrane's bias risk tool was used to evaluate the randomized controlled trials and make a risk bias map. Bias analysis included random sequence generation, random scheme concealment, participant blinding, result evaluation blinding, data integrity, selective reporting, and other biases. Each bias risk level was divided into low, high or unclear, and different color blocks represented the results. Two independent researchers conducted the quality assessment.

## 3. Results

### 3.1. Search Results and Research Characteristics

A total of 69232 documents were retrieved from different databases, of which 43486 duplicate documents were eliminated. The remaining literature were reviewed and evaluated according to the inclusion criteria, and 10 were finally selected. The specific inclusion and exclusion process is shown in Figure 1. Document characteristics and experimental result data were counted, and a quality review was conducted. See Table 1 for a summary of study characteristics and scores of the modified Jadad scale. A total of 523 Parkinson's disease patients with HY stages 1-3 were included in the study. Eligible research types included aerobic exercise, resistance exercise, and physical therapy-based multidisciplinary rehabilitation. The duration of physiotherapy varied from 6 months to 2 years. In addition, drug treatment status in different studies was also distinct. 6 of them were combined with drug treatment, while patients in 2 special studies took the drug part of the time, and the drug was stopped part of the time during the whole experiment (see Table 1 for detailed literature research characteristics).

### 3.2. Bias Risk and Literature Quality Assessment

Figure 2 is a summary of the bias risk of each literature, and Figure 3 is a bar chart of the bias risk of the included studies. Each study had its limitations or could not be judged. In other words, no investigation was completely low risk. All studies had a low risk of blinding or other bias in outcome assessment. In current meta-analysis, most included studies have low risk in random sequence generation, random scheme hiding, and data integrity. However, most studies had a bias in the blind method for participants, demonstrating a high risk. The improved Jadad scale is also a general tool to evaluate the quality of literature. The literature scores were distributed between 4 and 6, and most of the literature scores were 5. The included literature was of high quality. The studies included in this paper were heterogeneous, so funnel analysis was not applicable.

### 3.3. Effect of Long-Term Physical Therapy on Motor Symptoms of Patients with Combined Antiparkinson Drugs

395 patients in 7 RCT studies were included in the analysis [11–13, 21, 22, 25, 26]. During long-term physical therapy, the changes in the MDS-UPDRS motor score before and after using antiparkinson drugs were analyzed. Therefore, the impact of long-term physical therapy on motor symptoms of patients with antiparkinson drugs was evaluated (see Figure 4 for details). The total meta-analysis data are shown in Figure 4(a). The data showed that long-term physical therapy could improve patients' motor symptoms with combined antiparkinson drugs (SMD = −0.47, 95%CI = −0.83, − 0.12, Z = 2.61, *P* = 0.009). Meanwhile, I^2^ = 65% indicated significant heterogeneity among the studies. Further, the studies were divided into three types according to the type of physical therapy: aerobic exercise, resistance training, and physical therapy-based multidisciplinary rehabilitation. Subgroup analysis was conducted according to three types, as shown in Figure 4(b). The results failed to show statistically significant results (*Z* = 1.53, *P* = 0.13, *Z* = 1.28, *P* = 0.2, *Z* = 0.86, and *P* = 0.39). The subgroup of aerobic exercise and multidisciplinary rehabilitation group showed significant heterogeneity (I^2^ = 81% and I^2^ = 85%).

### 3.4. Effect of Long-Term Physical Therapy on Motor Symptoms of Patients without Antiparkinson Drugs

A total of 240 patients in 4 RCT studies were included in the analysis [21, 23–25]. The changes in MDS-UPDRS motor score before and after long-term physical therapy in patients who did not use antiparkinson drugs were analyzed. Therefore, the impact of long-term physical therapy on motor symptoms of patients who stopped using antiparkinson drugs was evaluated (see Figure 5 for details). The total meta-analysis data are shown in Figure 5(a). The data showed that long-term physical therapy significantly improved the motor symptoms of patients who stopped using antiparkinson drugs (SMD = −0.86, 95%CI = −1.47, − 0.24, *Z* = 2.73, and *P* = 0.006). Furthermore, I^2^ = 77% showed significant heterogeneity among the studies. Subgroup analysis of each study according to each physiotherapy type is shown in Figure 5(b). The multidisciplinary rehabilitation subgroup failed to show a significant positive effect, and the heterogeneity of this subgroup was high, I^2^ = 89%. Only one study was about the aerobic group and resistance training. Between them, resistance training showed a positive impact on improving exercise symptoms.

### 3.5. Effect of Long-Term Physical Therapy on Daily Activities (ADL) of Parkinson's Patients

A total of 474 patients in 9 RCT studies were included in the analysis [11–13, 20–24, 26]. The changes in MDS-UPDRS ADL scores before and after long-term physical therapy were analyzed to evaluate the impact of long-term physical therapy on the daily activities (ADL) of Parkinson's patients (see Figure 6 for details). The total meta-analysis data are shown in Figure 6(a). The data showed that long-term physical therapy had no significant effect on the daily activities (ADL) of Parkinson's patients (SMD = −0.31, 95%CI = −0.70, 0.08, *Z* = 1.54, and *P* = 0.12). In addition, I^2^ = 75% showed significant heterogeneity among the studies. Further subgroup analysis of each physiotherapy type is shown in Figure 6(b). The aerobic exercise and resistance training groups had no significant effect, but the multidisciplinary rehabilitation group showed positive improvement (SMD = −0.67, 95%CI = −1.32, − 0.03, *Z* = 2.04, and *P* = 0.04).

### 3.6. Effect of Long-Term Physical Therapy on Antiparkinson Drug Dosage (LED) of Parkinson's Patients

A total of 449 patients in 8 RCT studies were included in the analysis [11, 12, 20, 21, 24–26]. Since patients used different Parkinson's drugs, levodopa equivalent dose (LED) was used for unified analysis and measurement to analyze the changes in LED dosage before and after long-term physical therapy. Furthermore, the impact of long-term physical therapy on the antiparkinson drug dosage (LED) of Parkinson's patients was evaluated (see Figure 7 for details). The total meta-analysis data are shown in Figure 7(a). The data showed that long-term physical therapy could reduce the LED dose of Parkinson's patients and the difference was statistically significant (SMD = −0.45, 95%CI = −0.79, − 0.11, *Z* = 2.58, and *P* = 0.010). I^2^ = 67% showed significant heterogeneity among the studies. Further subgroup analysis of each physiotherapy type is shown in Figure 7(b). The aerobic exercise and resistance training groups had no significant effect, but the multidisciplinary rehabilitation group showed a positive impact (SMD = −0.68, 95%CI = −1.25, − 0.11, *Z* = 2.35, and *P* = 0.02).

## 4. Discussion

Currently, there are fewer systematic evaluations and meta-analyses to study the effects of long-term physical therapy on motor symptoms, quality of life, and dosage of antiparkinson drugs in patients with Parkinson's disease. Meanwhile, there is a lack of research evidence of high-quality literature analysis. This paper summarized and analyzed the impact of long-term physical therapy on the results of Parkinson's patients. We divided them into three groups according to the type of physical therapy. We classified and analyzed each subgroup to explore the impact of a specific kind of physical therapy on the results, thus seeking the best treatment type. The analysis results of this study demonstrated that physical therapy for at least 6 months or longer for patients with mild to moderate Parkinson's HY could effectively improve the motor symptoms of Parkinson's patients than the control group, mainly the short-term intervention group of physical therapy, other types of intervention group, or no treatment group, whether or not combined with antiparkinson drugs. Meanwhile, long-term physical therapy could reduce the LED dose of patients treated with drugs. Increasing literature emphasizes the importance of early long-term physical intervention for Parkinson's patients [27, 28], and the conclusion of this paper also supports this view. Although there is little research on long-term physical therapy, this paper still conducted a subgroup analysis according to the type of physical therapy. Among them, the multidisciplinary rehabilitation group showed that it could improve ADL and LED.

To investigate the effect of long-term physical therapy on motor symptoms of patients with combined antiparkinson drugs, we included 7 RCT studies. The analysis showed that long-term physical therapy combined with antiparkinson drugs could improve motor symptoms, and the difference was statistically significant. However, no statistically significant difference was found in each analysis subgroup. On the one hand, the methods of physical therapy were different, the treatment time was also different, and the heterogeneity of methodology was quite considerable, which caused variation in the result. On the other hand, due to the mixed use of antiparkinson drugs and the extended research time, it was difficult to analyze whether a specific intervention or the combined use of drugs and exercise was responsible for the result. Moreover, one of the literature included in this study showed a greater effect on improving medication status compared with other literature [26]. Still, other studies did not show significant statistical differences. This result should be carefully considered.

In this paper, 4 literatures were included to analyze the impact of long-term physical therapy on patients who stopped using antiparkinson drugs. The final summary analysis showed that long-term physical therapy had achieved the remission of motor symptoms. But in the subgroup analysis, only one resistance training had a statistically significant effect.

9 studies were included to analyze the effect of long-term physical therapy on daily activities (ADL) of Parkinson's patients. The results showed that there was no statistically significant effect. However, subgroup analysis showed that the multidisciplinary rehabilitation group showed positive improvement. Although the multidisciplinary therapy included in the literature mainly consisted of physical therapy, it also had some visual and auditory guidance training to improve gait and posture [24, 26]. Several RCT experiments showed that multidisciplinary rehabilitation therapy combined with gait and posture management could improve the daily life of Parkinson's patients [29, 30]. Their results also suggested that multidisciplinary therapy, such as physical therapy combined with posture and gait management, had a certain positive significance for improving ADL. In addition, the symptoms of Parkinson's patients also include non-motor symptoms, such as sleep disturbance, mood disorders, and autonomic dysfunction [2], which also widely affect the daily life of patients, and also cause the diversity of reasons for improving patients' daily life. A single change in a patient's motor symptoms was not completely effective in improving the patient's daily living score. The multidisciplinary rehabilitation treatment model has more treatment modes and improves the functional impairment of the patients more widely, which is also the potential reason why the multidisciplinary treatment mode improves the daily life score of Parkinson's patients.

A total of 8 articles were included in the analysis of the impact of long-term physical therapy on the LED dose. Although the research was heterogeneous, the summary analysis results suggested that it was positive and beneficial. However, the subgroup analysis of the five literatures showed that multidisciplinary rehabilitation had a statistically significant impact on ADL, indicating that long-term multidisciplinary rehabilitation based on physical therapy positively affected ADL. The result might suggest that multidisciplinary rehabilitation reduces the drug use of progressive Parkinson's patients.

The study also has limitations. This study mainly focused on a wide range of physical therapy measures and did not focus on a specific treatment type. Therefore, the number of studies of each intervention type was small, so the interpretation of the results of different intervention types was relatively weak. Secondly, low-quality studies and studies with an inaccuracy of medication status or score changes, studies with unknown status, or lack of mean and standard deviation were excluded to ensure the reliability of research evidence. However, this resulted in a small number of included literatures. In addition, some control groups in the included literature had some short-term physical interventions. Despite the intervention period, the bias caused by these control groups could not be excluded entirely.

The analysis results of this paper showed that physical therapy for at least 6 months or longer for patients with mild to moderate Parkinson's HY could effectively improve the motor symptoms of patients with Parkinson's disease, whether combined with antiparkinson drug therapy or not. Compared with the control group, that is, the short-term intervention group of physical therapy, other types of intervention group, or no treatment group, long-term physical therapy could reduce the LED dose of patients with drug therapy. The results of this study emphasized the importance of persisting in long-term physical therapy, regardless of whether it is in the state of drug treatment, and the necessity of continuous physical therapy from the early and middle stages of the disease [27]. The improvement can boost the confidence of Parkinson's patients and make them pay more attention to and adhere to long-term physical therapy. In addition, reducing drug dose can minimize the risk of exercise complications related to drug dose, thus helping reduce patients' relevant economic burden.

## Figures and Tables

**Figure 1:** Document screening and exclusion process.

**Figure 2:** Summary of study bias risk.

**Figure 3:** Study bias risk map.

**Figure 4:** Effect of long-term physical therapy on motor symptoms of patients with combined antiparkinson drugs. (a) Total meta-analysis data and (b) subgroup analysis data by physical therapy type.

**Figure 5:** Effect of long-term physical therapy on motor symptoms of patients without antiparkinson drugs. (a) Total meta-analysis data and (b) subgroup analysis data by physical therapy type.

**Figure 6:** Effect of long-term physical therapy on daily activities (ADL) of patients with Parkinson's disease. (a) Total meta-analysis data and (b) subgroup analysis data by physical therapy type.

**Figure 7:** Effect of long-term physical therapy on the dosage (LED) of antiparkinson drugs in patients with Parkinson's disease. (a) Total meta-analysis data and (b) subgroup analysis data by physical therapy type.

**Table 1:** Characteristics and quality scores of included literature.

Study	Subjects, *n*		HY stage	Intervention		Outcome measures	Medication state in evaluation time	M-Jadad scale
	Experimental group	Control group		Experimental group	Control group			
Au 2022 [11]	15	15	1-3	Multidisciplinary rehabilitation 6 months	Multidisciplinary rehabilitation 6 weeks	MDS- UPDRS motor, ADL LED, etc.	On	5
Yang 2022 [13]	30	30	1-3	Multidisciplinary rehabilitation 18 months	Multidisciplinary rehabilitation 4 months	MDS-UPDRS motor, ADL LED, etc.	On	5
Mak 2021 [12]	33	31	1-3	Aerobic exercise 6 months	Usual care 6 months	MDS-UPDRS motor, ADL LED, etc.	On	5
Tollar 2019 [20]	19	20	1-2	Multidisciplinary rehabilitation 2 years	No exercise 2 years	MDS-UPDRS ADL, LED, etc.	On	4
Kolk 2019 [21]	65	65	1-2	Aerobic exercise 6 months	Stretching and relaxation 6 months	MDS-UPDRS motor, ADL LED, etc.	On/off	6
Ferreira 2018 [22]	18	17	1-3	Resistance exercise 6 months	No intervention 6 months	MDS-UPDRS motor, ADL, etc.	On	5
Kolk 2018 [23]	22	15	1-2	Aerobic exercise 6 months	No intervention 6 months	MDS-UPDRS motor, ADL, etc.	Off	5
Frazzitta 2015 [24]	20	20	1-2	Multidisciplinary rehabilitation 2 years	Usual care 2 years	MDS-UPDRS motor, ADL LED, etc.	Off	5
Cocros 2013 [25]	20	18	1-3	Resistance exercise 1 year	Fitness count exercise 1 years	MDS-UPDRS motor, LED, etc	On/off	6
Frazzitta 2012 [24]	25	25	3	Multidisciplinary rehabilitation 1 year	Usual care 1 year	MDS-UPDRS motor, ADL, LED, etc	On	4

*N*: patients number; HY: Hoehn and Yahr stage; MDS-UPDRS: Movement Disorder Society-sponsored revision of the Unified Parkinson's Disease Rating Scale; ADL: activities of daily living scale; LED: levodopa equivalent dose; on: on medication state; off: off medication state. M-Jadad scale: modified Jadad scale.

## Data Availability

The data used to support the findings of this study are included within the article.
